RETRACTED

# Expression of PD-L1 and BRCA1 in Triple-Negative Breast Cancer Patients and Relationship with Clinicopathological Characteristics

**DOI:** 10.1155/2021/5314016

**Published:** 2021-10-22

**Authors:** Xianghua Huang, Xiangqian Wang, Hongyan Qian, Xiaoxia Jin, Guoqin Jiang

**Affiliations:** ^1^Department of General Surgery, The Second Affiliated Hospital of Soochow University, Suzhou 215004, Jiangsu, China; ^2^Department of Breast Surgery, Affiliated Tumor Hospital of Nantong University, Nantong 226321, Jiangsu, China; ^3^Department of Radiation Oncology, Affiliated Tumor Hospital of Nantong University, Nantong 226321, Jiangsu, China; ^4^Key Laboratory of Cancer Research Center Nantong, Tumor Hospital Affiliated to Nantong University, Nantong 226321, Jiangsu, China; ^5^Department of Pathology, Nantong Tumor Hospital, Affiliated Tumor Hospital of Nantong University, Nantong 226321, Jiangsu, China

## Abstract

**Objective:**

To study the expression of programmed cell death ligand-1 (PD-L1) and breast cancer susceptibility gene 1 (BRCA1) in triple-negative breast cancer (TNBC) patients and analyze their relationship with clinicopathological characteristics.

**Methods:**

76 TNBC tissues were collected as the research object, while 60 adjacent tissues were used as controls. All patients underwent surgical treatment, and the expression of PD-L1 and BRCA1 in cancer tissues and adjacent tissues was detected by immunohistochemistry. At the same time, the relationship between PD-L1, BRCA1, and clinicopathological characteristics of patients with TNBC (including patient age, menopausal status, tumor size, lymph node metastasis, histological grade, Ki-67 expression, and p53 expression) were analyzed by univariate and logistic multivariate analysis.

**Results:**

The positive expression rate of PD-L1 in the TNBC group was 64.47%, which was higher than the control group by 41.67%. The positive expression rate of BRCA1 was 27.63%, which was lower than the control group by 48.33%. PD-L1 expression has no significant relationship with age, menopausal status, and p53 expression in TNBC patients. TNBC patients with tumors ≥2 cm, histological grade III, lymph node metastasis, and Ki-67 expression ≥20% had higher PD-L1 positive expression rates. The tumor size, Ki-67 expression, and PD-L1 expression of TNBC patients have independent effects. The expression of BRCA1 has no significant relationship with menopausal status, tumor size, Ki-67 expression, etc. TNBC patients with age <45 years, histological grade I or II, no lymph node metastasis, and high p53 expression positive rate had higher BRCA1 positive expression rate. The age of TNBC patients, p53 expression, and BRCA1 expression have independent effects.

RETRACTED

**Conclusion:**

In TNBC cancer tissues, there is a high expression of PD-L1 and low expression of BRAC1. The tumor size, Ki-67 expression, and PD-L1 expression of TNBC patients have independent effects. The age of TNBC patients, p53 expression, and BRCA1 expression have independent effects.

## 1. Introduction

Triple negative breast cancer (TNBC) is a special type of breast cancer (BC) that refers to estrogen receptor (ER), progesterone receptor (PR), and human epidermal growth factor receptor. Human epidermal growth factor receptor 2 (HER2) is negatively expressed in BC, which is a highly heterogeneous tumor with biological characteristics such as strong invasiveness, high recurrence rate, and distant metastasis [1, 2]. In recent years, the field of cancer immunotherapy has become a research hotspot, especially for immune checkpoint targeted therapy, such as cytotoxic lymphocyte-associated antigen-4 (CTLA-4) and programmed death receptor-l (PD-1)/programmed death ligand-1 (PD-L1) axis, and breast cancer susceptibility gene 1 (BRCA1) [3]. PD-L1 is one of the main ligands of PD-1. It is highly expressed in the tumor microenvironment and can make tumor-related immune cells apoptosis and participate in cancer immune escape [4]. BRCA1 is an important tumor suppressor gene that can interact with oncogenes or tumor suppressor gene proteins, cell cycle regulatory proteins, DNA repair proteins, and other proteins to regulate the cell cycle and repair DNA damage [5]. TNBC has a poor overall prognosis and lacks effective therapeutic targets, so it is particularly important to explore the occurrence and development of TNBC [6]. In this study, by detecting the expression of PD-L1 and BRCA1 in TNBC pathological tissues and exploring their relationship with the clinicopathological characteristics of TNBC, it hopes to provide clinical evidence for TNBC immunotherapy. The detail information is as follows.

## 2. Materials and Methods

### 2.1. General Information

The tissue wax blocks of 76 patients who were operated on in our hospital from September 2016 to September 2019 and whose pathological examination results were TNBC were collected. At the same time, 60 cases of adjacent tissues (taken from the edge of the tumor ≥3 cm) were selected as controls. The average age of the patients was (45.46 ± 8.77) years; none of them received chemotherapy, radiotherapy, or biological immunotherapy before surgery; immunohistochemical tests showed that ER, PR, and HER2 were all negatively expressed. This study was approved by the medical ethics committee of our hospital, and the patients and their families signed informed consent.

### 2.2. Research Methods

Immunohistochemistry was used to detect the expression of PD-L1 and BRCA1 in tissue blocks. The immunohistochemistry kit was purchased from Beijing Boaosen Biotechnology Co., Ltd., and the experimental operation was carried out in strict accordance with the kit instructions. The staining results are read by 2 or more pathologists. PD-L1 positive expression standard: yellow or brown particles appear in the cell membrane or cytoplasm; BRCA1 positive expression standard: yellow or brown particles appear in the nucleus or part of the cytoplasm. For staining, it is 3 points for brown, 2 points for brown, 1 point for light yellow, and 0 points for no color development. The percentage of positive cells higher than 80% is 4 points, 51%∼80% is 3 points, 11%∼50% is 2 points, 0%∼10% is 1 point, and less than 10% is 0 points. The product of the staining score and the percentage of positive cells is the final score. The total score ≥4 is positive, and <4 is negative. Clinical data such as patient age, menopausal status, tumor size, lymph node metastasis, histological grade, Ki-67 expression, and p53 expression were collected (Ki-67 expression in the form of protein positive expression: divided into ≥20% and <20%; p53 expression in the form of positive expression and negative expression: the product of staining score and the percentage of positive cells is the final score, and the total score ≥4 is positive, <4 is negative).

RETRACTED

### 2.3. Statistical Methods

Use SPSS19.0 software for data processing, the enumeration data are represented by examples (%), and the comparison between groups is done by *χ*^2^ test. Multivariate analysis adopts the logistic proportional hazard regression model, and *P* < 0.05 indicates that the difference is statistically significant.

## 3. Results

### 3.1. Expression of PD-L1 and BRCA1 in TNBC

The results of immunohistochemical staining showed that the PD-L1 positive in the TNBC group was located in the cell membrane, which was brown or brownish (Figures 1(a) and 1(b)); BRCA1 positivity is located in the nucleus with brownish-yellow particles (Figures 1(c) and 1(d)). The results showed that the positive expression rate of PD-L1 in the TNBC group was 64.47% (49/76), which was higher than 41.67% (25/60) in the control group (*P* < 0.05), and the positive expression rate of BRCA1 was 27.63% (21/76), which was lower than 48.33% (29/60) of the control group (*P* < 0.05), as shown in Figures 2 and 3.

### 3.2. The Relationship between the Expression of PD-L1 and BRCA1 and the Clinical Characteristics of TNBC Patients

The results showed that there was no significant relationship between PD-L1 expression and patient age, menopausal status, p53 expression, etc., and the difference was not statistically significant (*P* > 0.05). The PD-L1 positive expression rate was higher in patients with tumor ≥2 cm, histological grade III, lymph node metastasis, and Ki-67 expression ≥20% (*P* < 0.05). The expression of BRCA1 had no significant relationship with the menopausal status, tumor size, Ki-67 expression, etc., and the difference was not statistically significant (*P* > 0.05). The BRCA1 positive expression rate was higher in patients who were younger than 45 years old, histological grade was I or II, had no lymph node metastasis, and had a high positive rate of p53 expression (*P* < 0.05) as shown in Table 1.

RETRACTED

### 3.3. Logistic Regression Analysis of PD-L1 and BRCA1 Expression and Clinical Case Characteristics of TNBC Patients

Logistic regression analysis showed that the tumor size, Ki-67 expression, and PD-L1 expression in TNBC patients had an independent influence (*P* < 0.05). The age, p53 expression, and BRCA1 expression of TNBC patients have independent influence relationships (*P* < 0.05) as shown in Table 2.

## 4. Discussion

BC seriously harms women's health, and the incidence rate is increasing year by year, showing a trend of younger age. In 2012 alone, the number of new BC cases reached 17 million, with a mortality rate of 3.06% [7, 8]. Because TNBC lacks the expression of ER, PR, and HER2 genes, compared with other BC types, it lacks corresponding therapeutic targets, is less sensitive to endocrine therapy, and has its unique biological characteristics, so the therapeutic effect is not good and patients' prognosis is poor [9]. In normal tissues, PD-L1 inhibits its function by binding to PD-1 on the surface of immune lymphocytes, thereby inducing apoptosis of activated immune lymphocytes. The activation of the PD-1/PD-L1 pathway helps to reduce the immune response zone. The damage that comes protects the body from autoimmune diseases [10]. BRCA1 is an important tumor suppressor gene. If it is mutated, the product it encodes will be changed and it will not be able to play the role of its tumor suppressor gene. BRCA1 can cause cell proliferation and cell cycle abnormalities and then participate in the occurrence and development of tumors [11].

Among the 76 cases of TNBC and 60 cases of the control group included in this study, the results of immunohistochemical staining showed that PD-L1 positive in TNBC patients was located in the cell membrane, which was brown or brownish”; BRCA1 positive is located in the nucleus, with brownish-yellow particles. The positive expression rate of PD-L1 in the TNBC group was 64.47%, which was higher than 41.67% in the control group; the positive expression rate of BRCA1 was 27.63%, which was lower than 48.33% of the control group. This is basically consistent with the reports of Barrett MT and Sun Xinxin [12, 13].

RETRACTED

The results of this study showed that PD-L1 expression has no significant relationship with TNBC patients' age, menopausal status, p53 expression, etc. PD-L1 patients present with tumors ≥2 cm, histological grade III, lymph node metastasis, and Ki-67 expression ≥20%. The positive expression rate is higher. Tumor size, Ki-67 expression, and PD-L1 expression in TNBC patients have an independent influence relationship. Similar results of Kurata et al. [14] and related research pointed out that PD-L1 is positively correlated with Ki-67 expression [15]. The expression of BRCA1 has no obvious relationship with menopausal status, tumor size, Ki-67 expression, and so on in TNBC patients. BRCA1 positive expression rate is higher in patients who are younger than 45 years old, histological grade is I or II, no lymph node metastasis, and the positive rate of p53 expression is high. The age, p53 expression, and BRCA1 expression of TNBC patients have independent influence relationships. Young TNBC patients have better physical functions, strong metabolism, larger breast glands, and faster tumor growth. Studies have shown that the expression of BRCA1 is negatively correlated with age, that is, the younger the age, the higher the expression of BRCA1 [16]. The tumor suppressor gene p53 has the functions of maintaining the integrity of the cell genome, repairing DNA damage, and regulating the cell cycle. BRCA1 can enhance the p53-dependent transcription by acting with the gene p53, and better exert its tumor suppressor effect, and there is a positive correlation between the expression of the two [17].

In summary, in the cancer tissues of TNBC patients, there is a high expression of PD-L1 and a low expression of BRAC1. PD-L1 was independently affected by tumor size and Ki-67 expression, and BRCA1 expression was influenced by age and p53 expression. Both PD-L1 and BRCA1 are related to the clinicopathology of TNBC patients, but whether there is a regulatory effect between the two and whether it affects the occurrence and progression of TNBC require further research and discussion in subsequent experiments.

## Figures and Tables

**Figure 1:** Immunohistochemical results of PD-L1 and BRCA1 expression in TNBC and control groups. (a) PD-L1 expression in breast tissue of the control group (SP × 400). (b) PD-L1 expression in breast tissue of the TNBC group (SP × 400); (c) BRCA1 expression in breast tissue of the control group (SP × 400). (d). BRCA1 expression in breast tissue of the TNBC group (SP × 400).

RETRACTED

**Figure 2:** Expression of PD-L1 in the TNBC group and control group.

**Figure 3:** xpression of BRCA1 in the TNBC group and control group.

**Table 1:** The relationship between the expression of PD-L1 and BRCA1 and the clinical characteristics of TNBC patients (*n*, %).

Factor	*n*	PD-L1 (+)	*χ* ^*2*^ value	*P* value	BRCA1 (+)	*χ* ^*2*^ value	*P* value
Age (year)			1.946	0.163		5.812	0.016
≥45	52	31 (59.61%)			10 (19.23%)		
<45	24	18 (75.00%)			11 (45.83%)		

Menopausal state			0.104	0.747		0.458	0.499
Yes	46	29 (63.04%)			14 (30.43%)		
No	30	20 (66.67%)			7 (23.33%)		

Tumor size (cm)			4.414	0.036		0.245	0.620
≥2	51	37 (72.55%)			15 (29.41%)		
<2	25	12 (48.00%)			6 (24.00%)		

Histological grade			8.732	0.003		7.833	0.005
I, II	28	24 (85.71%)			13 (46.43%)		
III	48	25 (52.08%)			8 (16.67%)		

Lymph node metastasis			11.644	0.001		5.140	0.023
Yes	34	29 (85.29%)			5 (14.71%)		
No	42	20 (47.62%)			16 (38.10%)		

Expression of Ki-67			10.294	0.001		0.076	0.783
≥20%	56	42 (75.00%)			15 (26.78%)		
<20%	20	7 (35.00%)			6 (30.00%)		

Expression of p53			0.314	0.575		5.323	0.021
Positive	54	34 (62.96%)			19 (35.19%)		
Negative	22	15 (68.18%)			2 (9.09%)		

**Table 2:** Logistic regression analysis of PD-L1 and BRCA1 expression and clinical case characteristics of TNBC patients.

	Influencing factors	OR	95% CI	*P*
PD-L1	Tumor size	3.816	6.473	0.002
	Histological grade	0.852	2.137	0.456
	Lymph node metastasis	1.492	2.924	0.285
	Ki-67 expression	6.478	12.945	0.010

BRCA1	Age	4.751	8.629	0.015
	Histological grade	0.966	2.358	0.375
	Lymph node metastasis	0.489	1.237	0.648
	Expression of p53	3.582	7.274	0.008

## Data Availability

The primary data used to support the results of this study are available upon reasonable request to the corresponding author.
